# Activation of Wnt/β-catenin signalling promotes mesenchymal stem cells to repair injured alveolar epithelium induced by lipopolysaccharide in mice

This article has been retracted.

**DOI:** 10.1186/s13287-015-0060-y

**Published:** 2015-04-11

**Authors:** Shi-xia Cai, Ai-ran Liu, Song Chen, Hong-li He, Qi-hong Chen, Jing-yuan Xu, Chun Pan, Yi Yang, Feng-mei Guo, Ying-zi Huang, Ling Liu, Hai-bo Qiu

**Affiliations:** Department of Critical Care Medicine, Zhong-da Hospital, School of Medicine, Southeast University, 87 Dingjiaqiao Road, Nanjing, 210009 People’s Republic of China; Department of Critical Care Medicine, The Affiliated Hospital of Qingdao University, 16 Jiangsu Road, Qingdao, 266003 People’s Republic of China; State Key Laboratory of Natural Medicines, School of Life Science and Technology, China Pharmaceutical University, 24 Tongjiaxiang, Nanjing, 210009 People’s Republic of China

## Abstract

**Introduction:**

Mesenchymal stem cells (MSCs) have potential for re-epithelization and recovery in acute respiratory distress syndrome (ARDS). In a previous *in vitro* study, the results showed that the canonical Wnt/β-catenin pathway promoted the differentiation of MSCs into type II alveolar epithelial cells, conferred resistance to oxidative stress, and promoted their migration, suggesting that the Wnt/β-catenin pathway might be one of the key mechanisms underling the therapeutic effect of mouse MSCs in ARDS.

**Methods:**

Mouse MSCs stable transfected with β-catenin or green fluorescent protein control were transplanted intratracheally into the ARDS mice induced by lipopolysaccharide. Lung tissue injury and repair assessment were examined using haematoxylin and eosin staining, lung injury scoring, Masson’s trichrome staining and fibrosis scoring. Homing and differentiation of mouse MSCs were assayed by labelling and tracing MSCs using NIR815 dye, immunofluorescent staining, and Western immunoblot analysis. The inflammation and permeability were evaluated by detecting the cytokine and protein measurements in bronchoalveolar lavage fluid using enzyme-linked immunosorbent assay.

**Results:**

In this study, β-catenin-overexpressing MSC engraftment led to more significant effects than the GFP controls, including the retention of the MSCs in the lung, differentiation into type II alveolar epithelial cells, improvement in alveolar epithelial permeability, and the pathologic impairment of the lung tissue.

**Conclusion:**

These results suggest that the activation of canonical Wnt/β-catenin pathway by mouse MSCs by overexpressing β-catenin could further improve the protection of mouse MSCs against epithelial impair and the therapeutic effects of mouse MSCs in ARDS mice.

## Introduction

Acute respiratory distress syndrome (ARDS) is the major cause of acute respiratory failure in critically ill patients, with a mortality as high as 40% despite improvements in supportive care [1,2]. The physiological hallmark of ARDS is the disruption of the alveolar-capillary membrane barrier, leading to development of noncardiogenic pulmonary oedema, in which a proteinaceous exudate floods the alveolar spaces, impairs gas exchange, and precipitates respiratory failure. Therefore, the repair and regeneration of the alveolar epithelium is associated with the treatment of ARDS [3].

Mesenchymal stem cells (MSCs), with their properties of multipotency and immunoregulation, are able to differentiate into alveolar epithelial cells, promote re-epithelialisation, alleviate inflammation, improve pathological impairment, and even reduce mortality in ARDS models [4-6]. However, the therapeutic effects remain limited because of the low engraftment and differentiation rates of MSCs in the lung tissue of ARDS models [7,8]. Therefore, clarifying the mechanisms underlying MSC function in epithelial repair in ARDS may lead to the improvement of cellular retention in injured lung tissue, differentiation of MSCs into alveolar epithelial cells and the MSC-mediated therapeutic effects in ARDS.

The canonical Wnt signalling pathway, which depends on the accumulation of β-catenin, is one of the fundamental pathways in cell proliferation and motility, cell fate decisions, cell polarity during embryonic development and adult tissue homeostasis [9]. Several recent studies have shown that Wnts and their downstream canonical signalling have critical effects on the self-renewal and differentiation of MSCs, which express a number of ligands, receptors, and inhibitors of the Wnt pathway [10].

In our previous study, we found that activation of the canonical Wnt/β-catenin pathway promotes the differentiation of mouse bone marrow-derived MSCs (mMSCs) into type II alveolar epithelial (AT II), confers resistance to oxidative stress, and promotes their migration to injured lung tissue *in vitro* [11]. However, the role of the Wnt/β-catenin pathway in the fate and therapeutic effect of MSCs in ARDS remains unexplored *in vivo,* where a more complicated environment and regulatory mechanisms different from the specific and limited cultural conditions of *in vitro* differentiation may affect the MSCs. In our previous study, a long-term, stable mMSC line modified with activated β-catenin was constructed using lentiviral vectors and confirmed to be able to activate the Wnt/β-catenin pathway, which could regulate the proliferation, migration and differentiation of the MSCs; this cell line is suitable for *in vivo* investigations [12]. The aim of our current study was to identify the effect of β-catenin overexpression on the repair of injured alveolar epithelium and its overall therapeutic effect in lipopolysaccharide (LPS)-induced ARDS mice.

## Materials and methods

### Mesenchymal stem cell transfection and culture

mMSCs derived from the bone marrow of C57BL/6 mice was obtained from Cyagen Biosciences, Inc. (Guangzhou, China). The details of the transfection of MSCs by lentivirus vectors were described in our previous work [12]. After transfection, mMSCs carrying an empty vector and enhanced green fluorescence protein (eGFP) (control mMSCs) or mMSCs carrying both the β-catenin gene and eGFP (mMSC-Ctnnb1) were cultured in a 1:1 mix of Dulbecco’s modified Eagle medium/nutrient mixture F-12 (Wisent, Inc., St-Bruno, Quebec, Canada) containing 10% foetal bovine serum (Wisent, Inc.) and 1% antibiotics (streptomycin and penicillin) and were incubated at 37°C in a humidified atmosphere of 5% CO_2_. The cells were used at passages 6 to 10 for the experiments.

### Preparation of experimental animals

Male C57BL/6 mice, aged 8 to 12 weeks and weighing 20 to 25 g, were obtained from the Laboratory Animal Center at the Academy of Military Medical Sciences (Beijing, China). All animal experiments performed in this study conformed to the Guide for the Care and Use of Laboratory Animals and were approved by the Institutional Animal Care and Use Committee.

### Murine model of lipopolysaccharide-induced acute respiratory distress syndrome

The mice were first anaesthetised with pentobarbital (50 mg/kg) by intra-peritoneal injection and received a single dose of LPS (100 μg intratracheally (i.t.)) from *Escherichia coli* serotype 0111:B4 (Sigma-Aldrich, St Louis, MO, USA) in 50 μl sterile normal saline (NS) [13]. The mice were then allowed to recover in a 100% oxygen chamber until fully awake. The control mice received 0.9% NS instead of LPS.

### Experimental protocol

The mice were randomly divided into four groups (n = 36 for each group): the NS + PBS group, in which mice received 30 μl phosphate-buffered saline (PBS) i.t. 4 hours after instillation of 0.9% NS i.t.; the LPS + PBS group, in which mice received 30 μl PBS i.t. 4 hours after the induction of ARDS; the LPS + mMSC control group, in which mice received control mMSCs (500,000 cells in 30 μl PBS) i.t. 4 hours after the induction of ARDS; and the LPS + mMSC-Ctnnb1 group, in which mice received mMSC-Ctnnb1 (500,000 cells in 30 μl PBS) i.t. 4 hours after the induction of ARDS. The mice were sacrificed after 3, 7 or 14 days, and samples were collected from each mouse for lung injury assessment, biochemical analysis, and histology. A diagram of the experimental protocol is shown in Figure 1.

**Figure 1:** Diagram of the experimental protocol. BALF, bronchoalveolar lavage fluid; i.t., intratracheally; LPS, lipopolysaccharide; mMSC, mouse mesenchymal stem cell; NS, normal saline; PBS, phosphate-buffered saline.

### Haematoxylin and eosin staining and lung injury scoring

The right upper lobe was embedded in paraffin and sagittally sliced at 5 μm. The sections were stained with haematoxylin and eosin. Oedema, alveolar and interstitial inflammation and haemorrhage, atelectasis, necrosis, and hyaline membrane formation were each scored using a 0 to 4 point scale (0, no injury; 1, injury in 25% of the field; 2, injury in 50%; 3, injury in 75%; and 4, injury throughout the field). The total lung injury score was calculated as the sum of these scores [14]. Ten randomly selected high-power fields (400×) in each slide were analysed by two investigators who were blinded to the mouse groups.

### Labelling and tracing of mesenchymal stem cells

The cultured control mMSCs and mMSC-Ctnnb1 were labelled with CellVue NIR815 dye (eBioscience Inc., San Diego, CA, USA) following the manufacturer’s instructions. NIR815-labelled cells (5 × 10^5^) were directly instilled into the trachea of the LPS + mMSC control and LPS + mMSC-Ctnnb1 mice. *Ex vivo* lungs from three subjects per group were imaged at three time points (3, 7 and 14 days post-instillation) using a Maestro *In-Vivo* Optical Imaging system (excitation = 786 nm, emission = 814 nm, exposition time 4,000 ms; Caliper Life Sciences, MA, Boston, USA) [15]. The autofluorescence spectra were then unmixed based on their spectral patterns using the Maestro 2.4 software (Caliper Life Sciences). The fluorescence intensity of the lungs was measured by placing the regions of interest on the organ, and the average signals were normalised based on the exposure time and the area of the region of interest (scaled counts/second).

### Immunofluorescent staining

Immunofluorescent staining for the detection of MSC engraftment homing and differentiation *in vivo* were performed as previously described [16]. Briefly, the left lung tissue samples from the LPS + mMSC control group and the LPS + mMSC-Ctnnb1 group were snap-frozen in liquid nitrogen then stored at −80°C until use. The tissue was embedded in optimal cutting temperature (Thermo Fisher Scientific, Bremen, Germany), and cut at a thickness of 10 μm. The slides were fixed in acetone at 4°C for 15 minutes and then blocked with 3% bovine serum albumin in PBS/0.3% Triton X-100 for 30 minutes at room temperature. After washing and draining, the slides were incubated overnight at 4°C with a green fluorescent protein (GFP) primary antibody (1:100, Abcam Incorporated, Cambridge, MA, USA) alone or with the same volume of GFP and pro-surfactant protein C (SP-C) primary antibodies (1:100, Santa Cruz Biotechnology, Paso Robles, CA, USA). After three washes with PBS, these slides were incubated with secondary Goat Anti-Mouse Alexa Fluor® 488 and Goat Anti-Rabbit Alexa Fluor® 647 antibodies (Abcam Incorporated) at a 1:200 dilution in 2% bovine serum albumin for 1 hour at 37°C in the dark. The nuclei were stained with DAPI for 5 minutes. The images were captured using a fluorescence microscope (Olympus, Tokyo, Japan). The retention or differentiation of transplanted MSCs was quantified based on the count of GFP-positive MSCs or the ratio of the count of GFP-positive to the count of SP-C-positive MSCs in randomly selected high-power fields (400×) for each slide by histopathologists blinded to the protocol design.

### Western immunoblot analysis

Total protein lysates were extracted using RIPA lysis buffer. The protein was separated by SDS-PAGE and electro-transferred to PVDF membranes (Millipore, Bedford, MA, USA). The membranes were blocked in Tris-buffered saline containing 0.1% Tween-20 and 5% bovine serum albumin for 1 hour at room temperature and then incubated at 4°C overnight with primary antibodies recognising SP-C, β-actin (Santa Cruz Biotechnology, Inc., Santa Cruz, CA, USA), or occludin (Abcam Incorporated). Immunoreactive bands were detected with chemiluminescence reagents (Thermo Fisher Scientific, Bremen, Germany).

### Cytokine and protein measurements in bronchoalveolar lavage fluid

Bronchoalveolar lavage fluid (BALF) was collected by flushing 1 ml ice-cold PBS back and forth three times through a tracheal cannula and then centrifuged at 800 g for 10 minutes. The concentrations of the interleukin (IL)-1β, IL-6 and IL-10 proteins in the supernatant were measured using murine cytokine-specific enzyme-linked immunosorbent assay (ELISA) kits (ExcellBio, Shanghai, China) strictly according to the manufacturer’s instructions. The amounts of total protein and albumin in the BALF were measured as a marker of epithelial permeability using ELISA kits (Cusabio Biotech, Wuhan, China). In addition, the levels of keratinocyte growth factor (KGF) in the BALF were measured using ELISA kits (Cusabio Biotech).

### Evaluation of the lung oedema

Lung oedema was evaluated using the ratio of lung wet weight to body weight (LWW/BW) measured as previously described [17]. Briefly, the whole lung was removed and cleared of all extrapulmonary tissues and the LWW/BW was calculated based on the values of lung wet weight and body weight (mg/g).

### Masson’s trichrome staining and fibrosis scoring

The lung sections were stained sequentially with Weigert’s iron haematoxylin solution, Biebrish scarlet-acid fuchsin solution, and aniline blue solution; a blue signal indicated positive staining for collagen. The criteria of Ashcroft were used [18], and lung fibrosis was quantified based on the findings in ten randomly selected high-power fields (400×) for each slide by histopathologists blinded to the protocol design.

### Statistical analysis

The data are presented as the means ± standard deviation. Statistical analyses were performed using SPSS 16.0 software package (SPSS Inc., Chicago, IL, USA). Comparisons among multiple groups were performed using one-way analysis of variance followed by Bonferroni’s *post-hoc* test if the data were normally distributed. A *P* value less than 0.05 was considered to be statistically significant.

## Results

### Effect of β-catenin-overexpressing mesenchymal stem cells on the pulmonary histopathology of lipopolysaccharide-induced acute respiratory distress syndrome mice

An increased thickening of the alveolar wall, alveolar and interstitial inflammatory cell infiltration, haemorrhaging, alveolar exudates, and oedema were found in the lung tissue of mice after LPS-induced lung injury, and the Smith score for quantification of the lung injury was also increased. However, these histopathologic characteristics and the Smith score were alleviated at 3, 7, and 14 days in the LPS + mMSC control and LPS + mMSC-Ctnnb1 groups compared with the LPS + PBS group (*P* < 0.05). The effect was greater in the LPS + mMSC-Ctnnb1 group than in the LPS + mMSC control group (*P* < 0.05) (Figure 2A,B).

**Figure 2:** Effect of control mouse mesenchymal stem cells (mMSCs) or β-catenin-overexpressing mMSCs on the histopathology of lipopolysaccharide (LPS)-induced lung injury and survival over 14 days. **(A)** Histopathological analysis of lung tissues from mice of all the experimental groups were performed at days 3, 7 and 14 after the LPS challenge (haematoxylin and eosin staining, magnification 200×). **(B)** Quantification of lung injury showed a significant reduction in the severity of lung injury in the LPS + mMSC control and LPS + mMSC-Ctnnb1 mice. The change was more significant in the LPS + mMSC-Ctnnb1 group than in the LPS + mMSC control group; n = 6 at each time point for each group. The results are expressed as the mean ± standard deviation. *P < 0.05, versus normal saline (NS) + phosphate-buffered saline (PBS) group; ^#^ *P* < 0.05, versus LPS + PBS group; ^&^ *P* < 0.05, versus LPS + mMSC control group.

### Overexpression of β-catenin increases the retention of mesenchymal stem cells in the lung after lipopolysaccharide challenge

*Ex vivo* NIR imaging was performed on the lungs from LPS + mMSC control and LPS + mMSC-Ctnnb1 mice 3, 7 and 14 days after MSC administration to trace the intrapulmonary mMSCs. Colour-coded fluorescence images indicated that the signals in the LPS + mMSC-Ctnnb1 group were stronger than those in the LPS + mMSC control group at the end of days 3, 7 and 14 after the LPS challenge. For each group, the signal gradually reduced after day 3. Though the signal decreased significantly on day 14 after the LPS challenge, it could still be detected (Figure 3A). Similar results were also observed using an immunofluorescent staining assay to detect the MSCs in lung tissue (Figure 3B).

**Figure 3:** Effect of β-catenin overexpression on the retention of mouse mesenchymal stem cells (mMSCs) in the lung after lipopolysaccharide (LPS) challenge. **(A)** *Ex vivo* NIR imaging of the lungs. Representative photographs of colour-coded fluorescence images are shown from three mouse lungs obtained 3, 7 and 14 days after mMSC administration from the LPS + mMSC control and LPS + mMSC-Ctnnb1 groups. **(B)** Immunofluorescent staining to detect mMSC engraftment in lung tissue is shown as green fluorescent protein (GFP)-positive (green; white arrows point to the GFP-positive cells). The nuclei were stained with DAPI (blue). Representative photographs are shown from six mouse lungs 3, 7 and 14 days after mMSC administration from the LPS+ mMSC control and LPS + mMSC-Ctnnb1 groups. All microphotographs were taken at 400× magnification (scale bar = 20 μm). The count of GFP-positive MSCs in randomly selected high-power fields (count/field) represent the mean ± standard deviation (n = 6). ^&^ *P* < 0.05, versus LPS + mMSC control group.

### Overexpression of β-catenin promotes the differentiation of mesenchymal stem cells into type II alveolar epithelial cells *in vivo*

Differentiation of the MSCs into AT II cells was evaluated 14 days after the MSC administration by analysing the expression of SP-C, a specific AT II cell marker, in the engrafted MSCs by immunofluorescence staining. Co-localisation of SP-C (red) and MSCs (green) in the lung tissue, which appeared yellow, could be seen in both the LPS + mMSC-Ctnnb1 and LPS + mMSC control groups; however, mMSC-Ctnnb1 treatment led to a higher differentiation efficiency of the MSCs into AT II cells than the control treatment (Figure 4A). The total expression of SP-C protein in the lung tissue 14 days after MSC administration was evaluated using Western blotting analysis. The results showed that SP-C protein was upregulated in the LPS + mMSC control group and the LPS + mMSC-Ctnnb1 group compared with the LPS + PBS group (*P* < 0.05), and the increase in the LPS + mMSC-Ctnnb1 group was more significant than the increase in the LPS + mMSC control group (*P* < 0.05) (Figure 4B).

**Figure 4:** Effect of β-catenin overexpression on the differentiation of mouse mesenchymal stem cells (mMSCs) into type II alveolar epithelial (AT II) cells *in vivo*. **(A)** The differentiation of mMSCs into AT II cells was detected by immunofluorescence staining 14 days after mMSC administration in mice from the lipopolysaccharide (LPS) + mMSC control and LPS + mMSC-Ctnnb1 groups. mMSC engraftment in lung tissue appears green fluorescent protein (GFP)-positive (green), a specific AT II cell marker pro-surfactant protein C (SP-C) appears red, and co-localisation in each case appears yellow (the white arrows point to double-positive cells). The nuclei were stained with DAPI (blue). All microphotographs were taken at 400× magnification (scale bar = 20 μm). The ratio of the count of GFP-positive to the count of SP-C-positive MSCs in randomly selected high-power fields is presented as mean ± standard deviation (n = 6). &*P* < 0.05 versus LPS + mMSC control group. **(B)** The expression of the SP-C protein in the lung tissue on day 14 after mMSC administration was evaluated using Western blotting analysis. β-actin was used as an internal control, and the results represent the mean ± standard deviation (n = 6). *P < 0.05 versus normal saline (NS) + phosphate-buffered saline (PBS) group; ^#^ *P* < 0.05, versus LPS + PBS group; ^&^ *P* < 0.05, versus LPS + mMSC control group.

### β-Catenin-overexpressing mesenchymal stem cells improved lipopolysaccharide-induced lung permeability

LWW/BW was calculated to evaluate lung oedema. LWW/BW was significantly reduced in the LPS + mMSC-Ctnnb1 group compared with the LPS + PBS group at days 3, 7 and 14 (*P* < 0.05) and in the LPS + mMSC control group at days 3 and 14 (*P* < 0.05). At day 14, LWW/BW was almost restored to normal levels in the LPS + mMSC-Ctnnb1 group (Figure 5A).

**Figure 5:** Effect of control mouse mesenchymal stem cells (mMSCs) or β-catenin-overexpressing mMSCs on lipopolysaccharide (LPS)-induced lung permeability. **(A)** Lung oedema was measured using the ratio of lung wet weight to body weight (LWW/BW). The results are shown for samples taken 3, 7 and 14 days after LPS exposure. **(B)** Total protein (TP) and **(C)** albumin (ALB) concentration in bronchoalveolar lavage fluid (BALF) were measured using mouse-specific enzyme-linked immunosorbent assays to evaluate the epithelial permeability of the lung. **(D)** Expression of the occludin protein in the lung tissue on day 14 after mMSC administration was evaluated using Western blotting analysis. β-actin was used as an internal control. **(E)** Keratinocyte growth factor (KGF) concentration in BALF was measured using a mouse-specific enzyme-linked immunosorbent assay. The data represent the mean ± standard deviation of six animals at each time point per group. *P < 0.05, versus normal saline (NS) + phosphate-buffered saline (PBS) group; ^#^ *P* < 0.05, versus LPS + PBS group; ^&^ *P* < 0.05, versus LPS+ mMSC control group).

To evaluate the effect of β-catenin-overexpressing MSCs on epithelial permeability of the lung, the total protein and albumin concentrations in the BALF were measured using mouse-specific ELISAs. Total protein and albumin were significantly reduced in the LPS + mMSC-Ctnnb1 group compared with the LPS + PBS group (*P* < 0.05) and the LPS + mMSC control group on days 3, 7 and 14 (*P* < 0.05). Significant decreases in total protein and albumin were also observed in the LPS + mMSC control group compared with the LPS + PBS group on days 3 and 7 (*P* < 0.05), while no difference was observed on day 14 (Figure 5B,C).

Additionally, to analyse the tight junctions of the pulmonary epithelial cells after MSC administration, occludin protein expression was evaluated in the lung tissue 14 days after MSC administration using Western blotting analysis. The results showed that occludin protein was upregulated in the LPS + mMSC control and LPS + mMSC-Ctnnb1 groups compared with the LPS + PBS group (*P* < 0.05), and the increase observed in the LPS + mMSC-Ctnnb1 group was more significant than that in the LPS + mMSC control group (*P* < 0.05) (Figure 5D).

The concentration of KGF, an important cytokine for the improvement of lung permeability, was measured in BALF using a mouse-specific ELISA. KGF was significantly increased in the LPS + PBS, LPS + mMSC control and LPS + mMSC-Ctnnb1 groups compared with the NS + PBS group on days 3, 7 and 14 (*P* < 0.05). Both control mMSC and mMSC-Ctnnb1 administration decreased the expression of KGF on day 3 compared with LPS + PBS treatment (*P* < 0.05). On day 14, KGF was higher in the LPS + mMSC-Ctnnb1 group than in the LPS + PBS (*P* < 0.05) and LPS + mMSC control groups (*P* < 0.05) (Figure 5E).

### β-Catenin-overexpressing mesenchymal stem cells attenuated acute lipopolysaccharide-induced pulmonary inflammation

The levels of the pro-inflammatory cytokines IL-1β and IL-6 and the anti-inflammatory cytokine IL-10 were measured in the BALF of mice 3 days after LPS treatment using ELISA. All three cytokines were significantly higher in the LPS + PBS group than in the NS + PBS group (*P* < 0.05). IL-1β and IL-6 were reduced in the LPS + mMSC control and LPS + mMSC-Ctnnb1 groups compared with the LPS + PBS group (Figure 6A,B), while IL-10 was increased (Figure 6C) (*P* < 0.05). Comparatively, the decrease in IL-1β and increase in IL-10 observed in the LPS + mMSC-Ctnnb1 group were more significant than the changes observed in the LPS + mMSC control group (*P* < 0.05).

**Figure 6:** Effect of control mouse mesenchymal stem cells (mMSCs) or mMSCs overexpressing β-catenin on acute lipopolysaccharide (LPS)-induced pulmonary inflammation. Levels of the proinflammatory cytokines **(A)** interleukin (IL)-1β, **(B)** IL-6 and anti-inflammatory cytokine **(C)** IL-10 in bronchoalveolar lavage fluid (BALF) in mice receiving MSCs at 3 days after LPS-induced acute respiratory distress syndrome were measured using enzyme-linked immunosorbent assay. Data are expressed as mean ± standard deviation (n = 6). *P < 0.05, versus normal saline (NS) + phosphate-buffered saline (PBS) group; ^#^ *P* < 0.05, versus LPS + PBS group; ^&^ *P* < 0.05, versus LPS+ mMSC control group.

### β-Catenin-overexpressing mesenchymal stem cells inhibited lung fibrosis

The deposition of collagen in lung tissue after 14 days of LPS exposure was evaluated by Masson’s trichrome staining and was markedly increased in the LPS + PBS, LPS + mMSC control and LPS + mMSC-Ctnnb1 groups compared with the NS + PBS group (*P* < 0.05). Reduced deposition of collagen was observed after intervention with either GFP-transfected MSCs or Ctnnb1-transfected MSCs when compared with LPS + PBS (*P* < 0.05), but the decrease observed in the LPS + mMSC-Ctnnb1 group was more significant than that observed in the LPS + mMSC control group (*P* < 0.05) (Figure 7).

**Figure 7:** Effect of control mouse mesenchymal stem cells (mMSCs) or mMSCs overexpressing β-catenin on lung fibrosis. **(A)** The lung fibrosis was evaluated by Masson’s trichrome staining 14 days after lipopolysaccharide (LPS) exposure (200×). **(B)** The quantification of lung fibrosis is shown as arbitrary units (n = 6). *P < 0.05, versus normal saline (NS) + phosphate-buffered saline (PBS) group; ^#^ *P* < 0.05, versus LPS + PBS group; ^&^ *P* < 0.05, versus LPS + mMSC control group.

## Discussion

MSCs have been shown to migrate to and engraft in injured lungs and differentiate into lung epithelial cells *in vivo* and have been considered to be a potential treatment for ARDS [4-6,19]. However, the relatively low engraftment and differentiation rate of MSCs in the injured lungs [4,7,8] limit their beneficial effects for ARDS therapy. In our previous *in vitro* study, we found that activation of the canonical Wnt/β-catenin pathway promoted the differentiation of mMSCs into AT II cells, migration to injured lung tissue, and resistance to oxidative stress [11]. This suggested that the canonical Wnt pathway may contribute to the improved therapeutic value of MSCs in ARDS. In the present study, we confirmed this positive effect of the Wnt/β-catenin pathway on LPS-induced ARDS mice using MSCs stably transfected with the β-catenin gene.

The canonical Wnt pathway is a fundamental regulatory pathway in development, differentiation, and other physiological functions of cells and organisms [9]. Canonical Wnt activation mainly depends on the accumulation of β-catenin. The binding of canonical Wnt ligands to the Frizzled (Fz) co-receptors and low-density lipoprotein receptor-related protein (LRP) 5 or 6 results in the inhibition of glycogen synthase kinase-3β (GSK-3β) and the accumulation of β-catenin, which then translocates into the nucleus to regulate target gene expression [20]. Therefore, β-catenin is considered to be the key signalling regulator of the canonical Wnt pathway. To obtain MSCs with stable, long-term transgene expression of β-catenin, lentiviral vectors were used for transfection in our study. According to our previous study, the lentiviral vector transduction efficiencies were as high as 95% even 20 passages after transduction, and the overexpression of β-catenin in the mMSCs led to the nuclear accumulation of β-catenin, suggesting increased activation of the Wnt/β-catenin pathway [12].

This construction of stable, long-term mMSCs lines with altered canonical Wnt signalling was also confirmed in our previous study by changes in cellular phenotype as well as altered biological behaviours including proliferation, differentiation, and migration of the mMSCs [12]. These characteristics suggested that the gene modification might facilitate ARDS therapy, and the observation that the administration of β-catenin-overexpressing mMSCs improved both the histopathological morphology and survival of ARDS mice more than treatment with mMSCs alone confirmed the benefits of β-catenin-overexpressing mMSCs for ARDS.

The biological functions of MSCs, including anti-inflammatory properties and abilities to differentiate into specialised cell types and mediate the repair of injured tissue, are based on their concentration and localisation in the injured or inflamed sites. Many studies have highlighted the ability of systemically or locally administered MSCs to migrate and home to inflamed, traumatised, ischaemic, and tumourous tissues [21-25] and their ability to specifically colonise the injured site, rather than intact loci [26]. Likewise, several studies have observed the enhanced recruitment of transplanted MSCs to the lung tissue in ARDS mice compared to normal control mice [5,27]. The positive effect of canonical Wnt/β-catenin signalling on the migration of MSCs has been demonstrated recently in other studies [28,29]. Our previous study also found that the migration of mMSCs to injured lung tissue through Transwell chambers was significantly enhanced when canonical Wnt signalling was stimulated by Wnt3a or LiCl [11]. In agreement with these studies, the results presented here show that β-catenin-overexpressing mMSCs exhibited increased retention in the lung of LPS-induced ARDS mice compared with control mMSCs.

In addition to the increased migration, the increased retention of MSCs in the lung tissue of ARDS mice may have a protective effect against adverse factors that decrease survival of the transplanted MSCs in complex *in vivo* situations, such as the production of oxidants, inflammatory factors, hypoxia, ischaemia, and so forth. In our previous study, we discovered that canonical Wnt signalling protected mMSCs against oxidative stress damage, which was evident by increased survival and inhibition of apoptosis [11], and that the β-catenin-overexpressing mMSCs exhibited increased proliferation compared with control MSCs *in vitro*. All of these mechanisms may contribute to the increased retention of mMSCs in the lung after LPS challenge.

AT II cells are characterised by their ability to synthesise and secrete alveolar surfactant that reduces surface tension and prevents collapse of the alveoli and by their ability to differentiate into type I alveolar epithelial cells that serve as progenitor cells for re-epithelialisation of impaired alveoli, significant in both physiological and pathological conditions [30]. The repair and regeneration of injured AT II cells is therefore critical for the recovery of patients with ARDS [31]. MSCs were proved in several investigations to be able to differentiate into AT II cells *in vivo* and *in vitro* [32,33]. Our previous study also demonstrated that canonical Wnt signalling is activated during the differentiation of mMSCs into AT II cells and that this enhanced signalling increases the expression of specific AT II cell markers [11]. Consistently, our present study showed that the activation of the canonical Wnt pathway through overexpression of β-catenin in mMSCs significantly increased their differentiation into AT II cells in the lung after LPS challenge.

Injury of the alveolar epithelium in ARDS is considered to be a key factor in the leakage of protein-rich oedema fluid into the interstitium and alveolar space [34]. Many studies have found that MSC treatment significantly reduces the lung wet-to-dry ratio, the amount of excess lung water, and the level of BALF protein, a marker of endothelial and epithelial permeability, in experimental ARDS [7,35]. In our study, we demonstrated that the β-catenin-overexpressing mMSCs also significantly improved the epithelial permeability, as evident from the LWW/BW, BALF albumin and total protein. It should be noted that the reduced total protein and albumin concentrations in the BALF is also attributed to the increased permeability of endothelium. As some studies found MSCs could preserve vascular endothelial integrity in the injured lungs after haemorrhagic shock [36], and even might differentiate into endothelial cells following bleomycin-induced lung injury [32], the effects of MSCs on the endothelial permeability in LPS-induced ARDS mice and whether β-catenin is involved in these effects is worth exploring in further studies.

The permeability barrier in the terminal airspace of the lung is due in a large part to tight junctions between alveolar epithelial cells [37]. Occludin is one of the well-characterised tight junction proteins and provides most of the barrier function of tight junctions [38]. Functional opening of the tight junction barrier and downregulation of occludin protein expression has been observed in acute lung injury in adult animals [39]. Our results presented here showed that the expression of occludin protein in the lung tissue was downregulated after LPS challenge and that mMSC treatment inhibited the repression of occludin protein. Moreover, the overexpression of β-catenin in mMSCs may provide additional benefits.

KGF, which is capable of stimulating proliferation and migration in AT II cells leading to the propagation of alveolar epithelial restitution [40] and reducing lung oedema and inflammation, was mechanistically implicated in the beneficial effect of MSCs on alveolar fluid clearance in ARDS. In our study, the results showed that treatment with β-catenin-overexpressing mMSCs markedly increased BALF KGF compared with treatment with mMSCs alone at day 14 after LPS instillation. These results indicated that the further improvement in lung permeability observed after treatment with β-catenin-overexpressing mMSCs may contribute to the repair of tight junctions and the increased paracrine signalling of KGF from the mMSCs.

MSCs can regulate the activity of a broad range of immune cells [41,42] and were found in several investigations, including the present study, to be able to inhibit inflammation in ARDS *in vivo*. Several lines of evidence supported this conclusion: pro-inflammatory cytokines such as interferon-γ, IL-1β, IL-6 were reduced, while the anti-inflammatory cytokine IL-10 was increased [7,27]. The overexpression of β-catenin in the mMSCs amplified this effect; however, the underlying mechanisms remain unclear and should be explored in the future.

In addition to the alveolar epithelial cells, engrafted MSCs in the lung could also differentiate into lung fibroblasts, myofibroblasts and interstitial monocytes, which may participate in pulmonary fibrosis [32]. The activation of Wnt/β-catenin signalling may be involved in the pulmonary fibrosis. Konigshoff and colleagues [43] demonstrated that dysregulation of Wnt/β-catenin signalling in AT II cells has been linked to the pathogenesis of pulmonary fibrosis. Moreover, Chilosi and colleagues [44] suggested that the aberrant nuclearisation of β-catenin in bronchiolar lesions could promote epithelial-mesenchymal transitions in the diseased lung. Another study found that β-catenin in the alveolar epithelium protected from lung fibrosis after intratracheal bleomycin [45]. Based on these observations, we evaluated whether the β-catenin-overexpressing mMSCs or control mMSCs alone increased the risk of pulmonary fibrosis after intratracheal LPS. The results of the present study showed that lung fibrosis decreased after treatment with control mMSCs alone and that this effect was more significant after the engraftment of β-catenin-overexpressing mMSCs.

## Conclusion

Activation of the canonical Wnt/β-catenin pathway through the overexpression of β-catenin increased the retention of mMSCs in the lung, promoted the differentiation of mMSCs into AT II cells, further improved the lung epithelial permeability, further attenuated acute pulmonary inflammation, and further inhibited lung fibrosis compared with control mMSCs, thus contributing to an improved therapeutic effect of mMSCs in ARDS.

## Abbreviations

ARDS: acute respiratory distress syndrome
AT II: type II alveolar epithelial
BALF: bronchoalveolar lavage fluid
BW: body weight
eGFP: enhanced green fluorescence protein
ELISA: enzyme linked immunosorbent assay
GFP: green fluorescent protein
i.t.: intratracheally
IL: interleukin
KGF: keratinocyte growth factor
LPS: lipopolysaccharide
LWW: lung wet weight
mMSC: mouse bone marrow-derived mesenchymal stem cell
MSC: mesenchymal stem cell
NS: normal saline
PBS: phosphate-buffered saline
SP-C: pro-surfactant protein C
